# Hybrid MWCNT and TiO_2_ Nanoparticle-Suspended Waste Tyre Oil Biodiesel for CI Engines

**DOI:** 10.1155/2023/8626155

**Published:** 2023-02-03

**Authors:** T. Sathish, V. Mohanavel, T. Raja, M. Ravichandran, P. Murugan, S. Suresh Kumar, Sultan Alqahtani, Sultan Alshehery, J. Isaac Joshua Ramesh Lalvani

**Affiliations:** ^1^Department of Mechanical Engineering, Saveetha School of Engineering, SIMATS, Chennai 602105, Tamil Nadu, India; ^2^Centre for Materials Engineering and Regenerative Medicine, Bharath Institute of Higher Education and Research, Chennai 600073, Tamil Nadu, India; ^3^Department of Mechanical Engineering, School of Technology, Glocal University, Delhi-Yamunotri Marg, Uttar Pradesh, 247121, India; ^4^Material Science Lab, Department of Prosthodontics, Saveetha Dental College and Hospitals, SIMATS University, Chennai 600077, Tamil Nadu, India; ^5^Department of Mechanical Engineering, K. Ramakrishnan College of Engineering, Trichy 621112, Tamil Nadu, India; ^6^Department of Mechanical Engineering and University Centre for Research & Development, Chandigarh University, Mohali 140413, Punjab, India; ^7^College of Engineering Mechanical Engineering Department, King Khalid University, Abha, Saudi Arabia; ^8^Department of Mechanical Engineering, Faculty of Mechanical and Production Engineering, AMIT, Arbaminch University, Ethiopia

## Abstract

Nowadays, scarcity arises in almost all our basic needs, including water, fuel, and food. Recycling used and scrapped things for a valuable commodity is highly appreciable for compensating for the globally fast-growing demand. This paper aims to investigate waste tyre oil for preparing biodiesel for CI engines by enhancing their performance with hybrid nanoparticles for preparing nanofuel and hybrid nanofuel. The nanoparticles (30–40 nm) of MWCNT and TiO_2_ were utilized to prepare nanofuels with nanoparticle concentrations of MWCNT (300 ppm) and TiO_2_ (300 ppm), respectively. In the case of hybrid nanofuel, the nanoparticle concentration of MWCNT (150 ppm) and TiO_2_ (150 ppm) was preferred. The performance of the proposed nanofuel and hybrid nanofuel with pure diesel was evaluated. The proposed fuel performance outperforms the combustion performance, has higher engine efficiency, and has fewer emissions. The best performances were noticed in hybrid nanofuel that has 32% higher brake thermal efficiency than diesel and 24% and 4% lower BSFC and peak pressure than diesel, respectively. The emission performance is also 29%, 50%, and 13% lower in CO, HC, and CO_2_ emissions than that in pure diesel.

## 1. Introduction

Energy and transformation of that energy is converted into its final form to meet our needs, such as for the generation of power or the movement of vehicles, etc. The IC engine plays a significant role in power generation and automotive vehicles. Accordingly, the alternate energy from the available resource within the country leads to developing self-satisfaction with the fuel for the IC engine. Kinds of research were focused on alternate fuels like fresh vegetable oil, used oils, and used wastes of different products. Basha et al. helped realize the alternate fuel production methods from various eatable and noneatable vegetables [1]. We investigated these kinds of new fuels individually. We blended them with the base diesel to identify their outcome concerning the IC engine in various load conditions and various operating conditions with different modifications in the engine number of research articles by multiple researchers. Ramadhas et al. conspicuously gave details regarding the favour of the vegetable oil using biodiesel conversion methods like transesterification, thermal cracking, and blending. They gave a clear impression of the different biodiesel production methods and their comparison, which is used to identify our approach concerning our oil consideration for the new investigation related to biodiesel [2]. Biodiesel was produced from some vegetable oils, such as camphor oil [3], neem oil, cashew nut oil [3], cottonseed oil [4, 5], castor oil [6], *Calophyllum* inophyllum [7], canola oil [8], and *Jatropha* oil [9], as well as from animal fatty oils, such as fish oil [10], chicken oil [11], pork skin oil [12], mutton fat oil [11], and beef fat oil [13]. In the same way, biodiesel can be derived by reusing or recycling of materials [14], For example, used cooking oil [15, 16], waste fishing net oil [17], waste plastics, and waste tyres [13, 18–21].

Among various wastes worldwide, tyre wastes of multiple vehicles are among the most critical pollutants. Every year, more than ten lakhs of tyres for use in automobiles are made worldwide [18]. India has six to seven percent of the share in waste tyres worldwide. For example, in 2016, only seven percent of waste tyres were recycled in the world, and the remaining ones were simply thrown as waste into landfills and sea. Nearly, 7650 lakhs of tyres were scrapped as waste. The pyrolysis process can use these waste tyres as fuel for IC engines. Pote and Patil studied the IC engine behaviour with waste tyre pyrolysis oil as a fuel. They compared different blendings like 10%, 25%, 50%, 60%, 75%, and 90% of waste tyre pyrolysis oil. The remaining volume is covered with the traditional diesel fuel in a high-speed VCR engine with eddy current loading. They concluded that the concentration of waste tyre pyrolysis oil is proportional to engine exhaust emissions like smoke, NOx and CO, but 10% of waste tyre pyrolysis oil with diesel blend produced better results for both performance and emissions [13].

Han et al. clearly explained the mechanism of tyre pyrolysis methods with a mass spectrometer containing a thermogravimetric analyzer. Four-step pyrolysis is recommended. Initially, up to 320°C, heating produces water vapourization and plasticizer decomposition. Second, further heating to 400°C leads to the deterioration of natural rubber in between these two steps. In the third step, up to 520°C, synthetic rubber corrosion occurs, and further heating produces a loss in weight. This is called the slow pyrolysis process [19]. Bhatt and Patel clearly explained the practicability of waste tyre pyrolysis oils into the CI engine as a fuel. Waste tyre pyrolysis oils can fuel industrial boilers and burning furnaces based on their excellent calorific value and low sulphur and ash concentration. However, in the IC engine, waste tyre pyrolysis oils are developed by increasing the quality of the fuel by blending the oil with the diesel fuel for better performance due to its slightly higher viscosity and density and less centre index than diesel fuel [20].

Vihar et al. employed waste tyre pyrolysis oil for the VCR engine with a turbocharger. They used the variable compression ratio, property enhancement methods, and pilot injections to obtain a similar diesel performance in the engine with various loading conditions. They suggested the waste tyre pyrolysis oil as the best substitute for the diesel in CI engines with turbochargers [21]. Yusof et al. reviewed different recent research articles related to the nanoparticle's influence on the outcome of the internal combustion engine with diesel fuel or biodiesel of vegetable oil or animal fatty oil, or synthetic oils. They mentioned the impact of individual metals (Si, Cu, Mg, Ni, and Zr), metal oxides (Fe_2_O_3_, Al_2_O_3,_ TiO_2_, MnO, CuO, AgO_2_, and CeO_2_), and nonmetals (GO, GNP, CNT, SWCNT, and MWCNT) on the engine fuel for the IC engine [22]. The nanoparticle size, concentration, quantity of mixing, and blending produced different results for engine outcomes. Senthil Kumar et al. investigated the influence of diesel fuel with titanium oxide (TiO_2_) nanoparticles in the two sizes such as 50 ppm and 100 ppm per lit of engine fuel water-cooledsingle-cylinder diesel engines. These variations provide enhancement in the calorific value (0.4 to 0.7%) and flash point (4.4 to 6.7%). Also, unburned hydrocarbon and NOx emissions were reduced by 1.7 to 2.3% and 3.7 to 4.1% compared with diesel fuel, respectively [23]. Similarly, smoke and CO get reduced in small amounts only. Nanthagopal et al. investigated the biodiesel of *Calophyllum inophyllum* with 50 ppm and 100 ppm of TiO_2_ and ZnO nanoparticle concentrations, respectively. These nanoparticle concentrations help increase thermal brake efficiency, decrease fuel consumption, and also reduce dangerous emissions like smoke emissions, NOx, CO, HC, and CO emissions in tailpipe exhaust [7]. Nithya et al. studied the biodiesel of canola with 300 ppm nanoparticle concentration of TiO_2_ in CI engine emissions. There is no mention of the engine's performance, but the authors only focused on emissions. 52% of smoke opacity, 30% of hydrocarbon, 32% of carbon monoxide, and 5% of NOx were reduced compared to diesel fuel emissions. At this point, NOx reduction is significantly less when compared to other emission reductions [8]. Hosseini et al. experimented with waste cooking oil and diesel blending (5% and 10% of biodiesel) in the addition of three different combinations of nanoparticle concentration such as 30 ppm, 60 ppm, and 90 ppm CNT in IC engines. The addition of the CNT into the engine fuel produces 3.67% greater power, 8.12% higher brake thermal efficiency, and 5.57% increased exhaust gas temperature but also helps reduce the fuel consumption and emissions of exhaust, except for nitrous oxides, compared to other emissions [15].

Sivathanu and Valai Anantham experimented with waste fishing net oil biodiesel mixed with the addition of MWCNT nanoparticles in the IC engine. It leads to less ignition delay, 3.83% increased brake thermal efficiency, and 3.8% less fuel consumption. From an emission point of view, 25% more secondary CO emission, 9% less UHC, 5% less NO, and 14.8% less smoke were obtained with 17.4% greater carbon dioxide emission. These variations were created with the impact of the MWCNT nanoparticle mixing into the fuel compared with the diesel fuel [17]. El-Seesy and Hassan dealt with the biodiesel of *Jatropha* oil with 50 ppm of three different nanoparticles like GO (graphene oxide), GNP (graphene nanoplatelet), and MWCNT (multiwalled carbon nanotube) in the IC engine as a fuel. MWCNT-mixed biodiesel produced 25% greater brake thermal efficiency and 35% less fuel consumption, and 15%, 45%, 55%, and 50% more secondary smoke emission, NOx emission, CO emission, and unburned hydrocarbon emission, respectively, than the remaining fuel in the same condition [9]. Sulochana and Bhatti focused on the biodiesel of waste fry oil with the addition of 25 ppm and 50 ppm MWCNT nanoparticle concentration comparison. They ensured that the nanoparticle's increase in the fuel leads to better performance and reduced emissions with less fuel consumption [16]. Hence, it is understood that the increase of nanoparticles like MWCNT improves fuel properties. In this study, we increased the nanoparticle contents in the fuel; specifically, waste tyre oil is an entirely new and novel investigation, which is focused in this investigation.

This investigation concentrated on increasing the output of the biodiesel of waste tyre pyrolysis oil (BWTPO) while using it in the compression ignition engine by adding nanoparticles. There are output (performance and exhaust emissions) comparisons between the nanoparticles of MWCNT and titanium oxide individually mixed with the 100% BWTPO fuel and both mixed nanoparticle combinations in the same fuel, and the schematic representation is shown in Figure 1.

## 2. Materials and Methods

This comparative investigation has four steps, which are as follows:

- Waste tyre pyrolysis oil extraction
- Nanofuel preparation
- Fuel characteristic measurement
- Testing on engines

### 2.1. Waste Tyre Pyrolysis Oil Extraction

Initially, used and scrapped tyres of different automotive vehicles were collected from other places of availability like mechanic shops, service centres, and waste collector shops. Then, the collected tyres were crushed up into pieces in the range of 0.02 to 0.025 cm. The flash pyrolysis method was implemented to extract the oil [24]. The solid setting time was less than 0.008 min, with a burning rate of more than 1200°C per second, and the temperature was maintained between 1000°C and 1300°C. This extraction method produced 78% of oil extraction, which can be obtained with 11% of char and 11% of gas.

The transesterification process occurs due to the reduced viscosity of pyrolysis oil. This oil was heated to 65°C with an agitator along with 200 ml per litre of methyl alcohol and 5 grams per litre of oil. These conditions were maintained for up to 90 minutes. Then, it was stored in a reverse conical-shaped vessel to separate glycerin from that by keeping it accessible at room temperature for one day. After that, the biodiesel of waste tyre pyrolysis oil (BWTPO shown in Figure 2) was separated from glycerin.

### 2.2. Nanofuel Preparation

In this investigation, there are three combinations of nanoparticles mixed with 100% of the biodiesel of the waste tyre pyrolysis oil. Nanofuel preparation is as follows:

1. BWTPO with MWCNT nanoparticle 300 ppm (BWTPO + MWCNT)
2. BWTPO with TiO_2_ nanoparticle 300 ppm (BWTPO + TiO_2_)
3. BWTPO with MWCNT nanoparticle 150 ppm and TiO_2_ nanoparticle 150 ppm (BWTPO + MWCNT and TiO_2_)
4. 100% of diesel
5. 100% of BWTPO

The considered nanoparticles were at 30 nm and had 180 W power. An ultrasonicator was used to mix the nanoparticles with an agitator.

The first nanofuel contains 300 ppm of MWCNT nanoparticles (shown in Figure 3(a)), the second nanofuel contains 300 ppm of TiO_2_ nanoparticles (shown in Figure 3(b)), and the third nanofuel contains 150 ppm of MWCNT nanoparticles and 150 ppm of TiO_2_ nanoparticles. These mixings were created with an ultrasonicator. The considered fuel properties are measured and tabulated in Table 1.

### 2.3. Combustion, Performance, and Emission Testing

These three nanoparticle-mixed fuels and 100% biodiesel and diesel fuel were tested with single-cylinder, four-stroke, variable compression ratio engines with a power of 3.5 kW at 1500 rpm. Loading is performed with the eddy current type, and cooling is performed with water. Flow sensors were fixed for air and fuel, and feedback and control were connected with the data acquisition system. The pressure transducer measured internal combustion pressure. The exhaust gases were analyzed by using an AVL gas analyzer and a smoke meter. These complete systems are shown in Figure 4 in a transparent manner.

## 3. Results and Discussion

### 3.1. Engine Performance by Nanofuels and Hybrid Nanofuels

Figure 5 clearly explains the relationship between the thermal brake efficiency and load variation from 20% to 100%. Diesel has 29% BTE in full-load conditions. Compared with diesel fuel, BWTPO, BWTPO + MWCNT, BWTPO + TiO_2_, and BWTPO + MWCNT and TiO_2_ have 10%, 25%, 21%, and 32% more brake thermal efficiency, respectively. Similarly, compared with biodiesel of waste tyre pyrolysis oil, nanofluids such as BWTPO + MWCNT, BWTPO + TiO_2_, and BWTPO + MWCNT & TiO_2_ have 13%, 10%, and 20% more brake thermal efficiency, respectively. BTE rises progressively for load variations because of changes in the calorific value with a concentration of the nanoparticle. Individual nanoparticle results were less than those of the combination of both nanoparticles. Mixed nanofuel produces higher BTE because of its high oxidation quality, which increases the engine's output with varying loads [7–9, 13, 15–17, 19–24].

### 3.2. Fuel Consumption Performance by Nanofuels and Hybrid Nanofuels

Various percentages of load-related specific fuel consumption correlations are mentioned in Figure 6 in a line diagram. This figure shows a reduction in fuel consumption by increasing the load for all fuels in this investigation. Among them, diesel and BWTPO have 0.8 kg/kW·hr and 0.7 kg/kW·hr specific fuel consumption in full-load conditions, respectively. BWTPO, BWTPO + MWCNT, BWTPO + TiO_2_, and BWTPO + MWCNT and TiO_2_, respectively, have 13%, 21%, 19%, and 24% less brake-specific fuel consumption than diesel fuel in full-load conditions. Likewise, BWTPO + MWCNT, BWTPO + TiO_2_, and BWTPO + MWCNT and TiO_2_, respectively, have 10%, 7%, and 13% lower BSFC than biodiesel of waste tyre pyrolysis oil. The speed of the engine leads to a reduction in fuel consumption [13, 19, 20]. Also, the nanoparticle concentration involves complete combustion, so it will help reduce fuel consumption [7–9, 15–17, 24].

### 3.3. CO Emission Performance by Nanofuels and Hybrid Nanofuels

Figure 7 shows the measured results of carbon monoxide emissions in a bar chart. Under varying load conditions, initially, all the fuels had more CO emission than diesel fuel at 25% of load conditions. In full-load conditions, 20%, 26%, 24%, and 29% less CO emissions were obtained by BWTPO, BWTPO + MWCNT, BWTPO + TiO_2_, and BWTPO + MWCNT and TiO_2_ fuels, respectively, when compared with diesel fuel. In the same way, BWTPO + MWCNT, BWTPO + TiO_2_, and BWTPO + MWCNT and TiO_2_ fuels, respectively, have 8%, 5%, and 11% less CO emissions than biodiesel of waste tyre pyrolysis oil. This dissimilarity is due to the maximum oxygen content available in the fuel [13, 19–22]. Oxidation in the fuel was created by the nanoparticles' individual and combined concentrations in the fuel [7–9, 15–17, 23, 24].

### 3.4. HC Emission Performance by Nanofuels and Hybrid Nanofuels

Figure 8 shows the relationship between unburned hydrocarbon emissions and load variations. From this comparison, diesel produces more HC emissions in all loading conditions than fuels. In full-load conditions, diesel fuel has an HC emission of 12 ppm. However, BWTPO, BWTPO + MWCNT, BWTPO + TiO_2_, and BWTPO + MWCNT and TiO_2_ fuels, respectively, have 42%, 45%, 48%, and 50% less unburned hydrocarbon emissions than diesel fuel in full-load conditions. At the same time, BWTPO + MWCNT, BWTPO + TiO_2_, and BWTPO + MWCNT and TiO_2_ fuels, respectively, have 5%, 10%, and 15% less HC emissions than the biodiesel of waste tyre pyrolysis oil. These HC emission differences were formed because of greater oxygen content availability [13, 19–22] in fuel and nanoparticle oxidation capacity [7–9, 15–17, 23, 24] than in diesel, which helps in maximum combustion. This will help reduce HC emissions more than diesel fuel does.

### 3.5. CO_2_ Emission Performance by Nanofuels and Hybrid Nanofuels

Carbon dioxide is the desirable pollutant in exhaust emissions compared to remaining emissions. Their relationship with various loads is mentioned in Figure 9. Diesel fuel has 1.80% carbon dioxide emission in full-load conditions. However, BWTPO, BWTPO + MWCNT, BWTPO + TiO_2_, and BWTPO + MWCNT and TiO_2_ fuels, respectively, have 33%, 20%, 17%, and 13% less carbon dioxide emissions than diesel fuel in full-load conditions. In the same conditions, BWTPO + MWCNT, BWTPO + TiO_2_, and BWTPO + MWCNT and TiO_2_ fuels, respectively, have 20%, 25%, and 30% more carbon dioxide emissions than the biodiesel of waste tyre pyrolysis oil. Complete combustion created by these differences leads to an increase in carbon dioxide emissions in fuels [7–9, 15–17, 22–24].

### 3.6. NOx Emission Performance by Nanofuels and Hybrid Nanofuels

In the same way, Figure 10 shows NOx emissions related to load variations.

Diesel fuel has a NOx emission of 350 ppm in full-load conditions. 17%, 8%, 11%, and 4% more NOx emissions were obtained by BWTPO, BWTPO + MWCNT, BWTPO + TiO_2_, and BWTPO + MWCNT and TiO_2_ fuels than that obtained by diesel fuel. However, compared with those of biodiesel of waste tyre pyrolysis oil, NOx emissions of 8%, 5%, and 11% reductions were obtained by BWTPO + MWCNT, BWTPO + TiO_2_, and BWTPO + MWCNT and TiO_2_ fuels, respectively. Combustion leads to a temperature rise in the engine, which increases NOx emissions [13, 19–22], but the nanoparticle concentration helps reduce the increase in NOx emissions [7–9, 15–17, 23, 24].

### 3.7. Combustion Performance by Nanofuels and Hybrid Nanofuels

Figure 11 shows variations of the peak pressure created during the combustion process concerning different load conditions. The diesel fuel reached 72 bars of the peak pressure, nearly equal to the BWTPO + MWCNT fuel's peak pressure. BWTPO and BWTPO + TiO_2_, respectively, have 8% and 3% higher peak pressure and BWTPO + MWCNT and TiO_2_ fuels have 4% lower peak pressure than diesel fuel in full-load conditions. However, BWTPO + MWCNT, BWTPO + TiO_2_, and BWTPO + MWCNT and TiO_2_, respectively, have 8%, 5%, and 11% lower peck pressure than the biodiesel of waste tyre pyrolysis oil. The peak pressure variation depends on the fuel's quality [13, 19–22]. The nanoparticle oxidation capacity helps create better combustion and reduces the peak pressure [7–9, 15–17, 23, 24].

Hence, in this investigation, alternate fuels like BWTPO with MWCNT nanoparticles of 300 ppm (BWTPO + MWCNT), BWTPO with TiO_2_ nanoparticles of 300 ppm (BWTPO + TiO_2_), BWTPO with MWCNT nanoparticles of 150 ppm and TiO_2_ nanoparticles of 150 ppm (BWTPO + MWCNT and TiO_2_), and 100% of BWTPO were prepared and characterized for fuel properties to ensure the fuel for supply and energy requirements (Table 1), and high cetane numbers 58 and 59 were found in nanofuels and hybrid nanofuels, respectively [25–28]. The engine performance of nanofuels and hybrid nanofuels is as follows: BWTPO + MWCNT, BWTPO + TiO_2_, and BWTPO + MWCNT and TiO_2_ have 13%, 10%, and 20% more brake thermal efficiency, respectively. The fuel consumption performance of nanofuels and hybrid nanofuels is as follows: BWTPO, BWTPO + MWCNT, BWTPO + TiO_2_, and BWTPO + MWCNT and TiO_2_, respectively, have 13%, 21%, 19%, and 24% less brake-specific fuel consumption than diesel fuel in full-load conditions [29]. The emission performance of nanofuels and hybrid nanofuels is as follows: In full-load conditions, 20%, 26%, 24%, and 29% less CO emissions were obtained by BWTPO, BWTPO + MWCNT, BWTPO + TiO_2_, and BWTPO + MWCNT and TiO_2_ fuels, respectively, when compared with diesel fuel. BWTPO, BWTPO + MWCNT, BWTPO + TiO_2_, and BWTPO + MWCNT and TiO_2_ fuels, respectively, have 42%, 45%, 48%, and 50% less unburned hydrocarbon emissions than diesel fuel in full-load conditions [30]. BWTPO, BWTPO + MWCNT, BWTPO + TiO_2_, and BWTPO + MWCNT and TiO_2_ fuels, respectively, have 33%, 20%, 17%, and 13% less carbon dioxide emissions than diesel fuel in full-load conditions [31]. The combustion performance of nanofuels and hybrid nanofuels is as follows: The diesel fuel reached a peak pressure of 72 bar, nearly equal to the BWTPO + MWCNT fuel's peak pressure. BWTPO and BWTPO + TiO_2_, respectively, have 8% and 3% higher peak pressure and BWTPO + MWCNT and TiO_2_ fuels have 4% lower peak pressure than diesel fuel in full-load conditions [32]. From the above results, it is understood that nanofuels and hybrid nanofuels performed well than diesel, in which hybrid nanofuels can be given top priority.

## 4. Conclusions

Generating nanofuels and hybrid nanofuels using waste tyre oil for CI engines with the help of MWCNT and TiO_2_ nanoparticles was discussed. The prepared fuels were tested, and the results were analyzed well. The following is the summary of this piece of research:

(i) Possibilities of biofuel production from waste tyre materials are discussed.
(ii) Biodiesel of waste tyre pyrolysis oil has better performance than diesel fuel in combustion and engine performance, but it causes higher exhaust emissions of HC, CO, and NOx, and MWCNT and TiO_2_ nanoparticle suspension decreased the same significantly.
(iii) Compared to individual fuel, a combination of the MWCNT and TiO_2_ nanoparticle-mixed biodiesel of waste tyre oil has better performance and less emission than BWTPO fuel. Based on diesel fuel, it has the following properties:
  - 32% more BTE
  - 24% and 4% lower BSFC and peak pressure
  - 29%, 50%, and 13% more secondary CO, HC, and CO_2_ emissions
  - 4% higher NOx emissions
(iv) So BWTPO + MWCNT and TiO_2_ fuels are the best alternative fuel for diesel in the CI engine.

This investigation selectively used MWCNT and TiO_2_ nanoparticles for enhancing waste tyre oil fuel for diesel engines and found that hybrid nanofuels outperformed diesel, waste tyre oil biodiesel, and also nanofuels. The investigation may be extended to hybrid nanofuels with the use of some other combinations more than two kinds [33].

## Figures and Tables

**Figure 1:** Schematic representation of this study.

**Figure 2:** Biodiesel of waste tyre pyrolysis oil.

**Figure 3:** Nanoparticles of (a) MWCNT and (b) TiO_2_.

**Figure 4:** Experimental setup.

**Figure 5:** Efficiency profile of diesel engines when using different fuels at different loads.

**Figure 6:** Relationship between specific fuel consumption (kg/kW·hr) and load variations (%).

**Figure 7:** Relationship between CO emission (%) and load variations (%).

**Figure 8:** Relationship between HC emissions (ppm) and load variations (%).

**Figure 9:** Relationship between carbon dioxide emissions (%) and load variations (%).

**Figure 10:** Relationship between NOx (ppm) and load variations (%).

**Figure 11:** Relationship between the peak pressure (bar) and load variations (%).

**Table 1:** Properties of the fuels.

Fuel/properties	Calorific value (kJ/kg)	Kinematic viscosity cSt @ 40°C	Density (kg/m^3^)	Flash point (°C)	Cetane number	Fire point (°C)
Diesel	44050	3.15	815	46	50	54
BWTPO	42800	3.72	905	24	56	33
BWTPO + MWCNT	44726	3.89	946	28	59	37
BWTPO + TiO_2_	44384	3.86	938	29	58	38
BWTPO + MWCNT and TiO_2_	45026	3.91	952	26	59	35

## Data Availability

The data used to support the findings of this study are included within the article and further data or information can be obtained from the corresponding author upon request.

## Abbreviations

BWTPO: Biodiesel of waste tyre pyrolysis oil
TPO: Tyre pyrolysis oil
GO: Graphene oxide
GNP: Graphene nanoplatelet
CNT: Carbon nanotube
SWCNT: Single-walled carbon nanotube
MWCNT: Multiwalled carbon nanotube
MnO: Manganese oxide
ZnO: Zinc oxide
CeO_2_: Cerium oxide
TiO_2_: Titanium oxide
Al_2_O_3_: Aluminium oxide
AgO_2_: Silver oxide
Ni: Nickel
Cu: Copper
Zr: Zirconium
NP: Nanoparticle
BTE: Brake thermal efficiency
BSEC: Brake-specific energy consumption
BSFC: Brake-specific fuel consumption
VCR: Variable compression ratio
EGT: Exhaust gas temperature
EGR: Exhaust gas recirculation
P: Pressure (bar)
ICP: Inner cylinder pressure
HC: Hydrocarbon
CO: Carbon monoxide
CO_2_: Carbon dioxide
NOx: Nitrous oxide
ppm: Parts per million
IC: Internal combustion
°C: Degree centigrade
Fe_2_O_3_: Ferric oxide.
